The article "Construction of Bilingual Teaching Mode Based on Digital Twinning Technology" was retracted in 2023. Reasons: signs of a paper mill; suspected computer-generated content; unreliable results or conclusions; lack of ethics approval or compliance.

# Construction of Bilingual Teaching Mode Based on Digital Twinning Technology

**DOI:** 10.1155/2022/9003806

**Published:** 2022-07-05

**Authors:** Jinming Cui

**Affiliations:** Center for Humanities and Social Sciences/School of Chinese studies, Xi'an International Studies University, Xi'an 710061, China

## Abstract

Based on the digital twin technology, a digital twin platform can be built to connect the real teaching space with the virtual teaching space and become the mainstream of online teaching space. All this has determined that the social demand for designers' education is undergoing fundamental changes. The so-called “scientific and technological progress, education first” bilingual education is undergoing comprehensive and profound changes in the digital age, which has a strong impact on the traditional bilingual teaching mode and concept. Traditional concepts, aging theoretical knowledge, and backward teaching methods will inevitably be eliminated and updated gradually in the contest with digitalization, which makes it necessary to transform traditional bilingual education into digital bilingual education. Through the comparative experimental analysis of the teaching effect, the independent sample *t*-test shows that the *t*-statistic is 3.634, and the corresponding significance level is 0.013, which is less than 0.05. It shows that there are significant differences between boys and girls in bilingual teaching in this class of digital twin technology experimental teaching. However, compared with the control class, the results of both boys and girls are higher, so to some extent, it shows that the application of digital twin technology experimental teaching in bilingual teaching will indeed produce certain results.

## 1. Introduction

In a bilingual classroom, teachers are the teaching subjects and students are the teaching objects. The amount of professional knowledge, teaching ability, and teachers' ability to express professional knowledge fluently and clearly in English directly affect the teaching effect. Whether students' professional vocabulary, listening, and speaking ability can perform well in bilingual classes will affect the teaching effect. Teachers impart knowledge to students through specific means, and the medium is textbooks. In the system theory, according to the principle of combining the human brain with the computer, the teaching methods adopted should be multimedia and writing on the blackboard. Using multimedia can free up the classroom capacity, and it is possible for specific writing on the blackboard to help students understand the content [1]. It is hard to describe. A good educational environment provides an atmosphere of teaching and learning for teachers and students. The environment here includes a classroom teaching environment and an extracurricular environment. The classroom environment mainly refers to the seamless communication channel between teachers and students, while the extracurricular environment mainly refers to bilingual culture, bilingual activities, and bilingual competitions provided by schools for students' bilingual education. Students always improve their bilingual skills by accepting bilingualism in a bilingual environment [2]. Teachers should adopt specific and appropriate teaching methods to create a good bilingual classroom environment. This means that students gain professional knowledge while improving their overall skills. Therefore, they complement each other. Without any element, the whole bilingual education system can hardly show a good educational effect.

This paper begins with the implementation of information technology integration in bilingual teaching and concludes with a quantitative analysis of the effect, in order to provide a reference for research into the theory and practice of information technology integration in bilingual teaching, to fully exploit the benefits of information technology, to serve bilingual teaching, to promote the application of information technology in bilingual teaching, and to promote the classification of information technology in bilingual teaching. Traditional classroom teaching prioritizes the selection of teaching methods, and there is usually a set number of what type of class, what kind of knowledge points, and what kind of teaching methods are required. The new geography teaching method, for example, is widely used: geography review class, which is primarily based on picture reading [3]. There are fewer rules and regulations on these choices in bilingual classes. Any teaching method that is conducive to improving students' learning quality and classroom teaching effect is acceptable in a bilingual class [4]. Bilingual classes, for example, can be combined with a guidance plan that can be used to assess students' self-study effect prior to class and guide class discussion. The essence of a bilingual classroom will not be altered by teachers' targeted instruction. The goal of implementing bilingual classrooms is to shift classroom instruction away from teacher-centered instruction and toward student-centered learning. As a result, teaching methods can be varied, which is a traditional classroom innovation and inheritance.

The digital platform is reshaping our teaching perception and experience, and it is also changing our way of thinking to solve problems. It realizes the subversive change of online teaching with full data drive, full field quantification, and full data visualization. Digital platform is an important means of online immersion teaching innovation in the process of teaching informatization, and it is also an important innovative application of Big Data + AI” [5, 6] in online teaching reform. In the experimental course of “Big Data and Smart Logistics” [7], we initially constructed an online immersion teaching system based on digital twin platform and designed the specific teaching process by using digital twin technology. Of course, this is only our preliminary exploration in the field of digital twinning and wisdom teaching. On the one hand, the digital platform can improve students' online learning enthusiasm through multisource data fusion. On the other hand, the digital twin platform can also deeply depict students' expressions and movements, intelligently identify students' individual needs, and make online immersion teaching truly teach students in accordance with their aptitude. Therefore, the digital twin platform will further guide online teaching toward digitalization, materialization, and intelligence in the future. Naturally, this innovative application and development will form a new form of classroom interaction based on big data, lead a new round of classroom teaching reform, and then influence the innovation and remodeling of modern education system [8].

The novelty of this paper is that it emphasizes the importance of bilingual teaching content and develops teaching design using various experimental teaching methods. Then, using two types of experimental teaching methods, students are tested using the compiled two-stage test questions as detection tools. The value of SOLO classification theory is then deconstructed, the test results are coded and assigned using SOLO classification theory, and the data is processed and analyzed to determine the difference in influence between digital experimental teaching and traditional experimental teaching on students' construction of bilingual teaching content. Finally, the research outlook is presented based on broad conclusions.

## 2. Related Work

In order to meet the arrival of international science and technology, information environment, and global economy, talents in the new century must face the standards of globalization, internationalization, and information in terms of language, culture, knowledge, and career. Therefore, in the training of talents in the new century, schools must conform to the needs of the times and intensify educational reform. The proposal and implementation of bilingual teaching is an important measure to truly change the traditional education system and establish new scientific education goals.

Gen-He H *E* E thinks that a general system is composed of multiple elements, and different elements of the same system are interrelated and interact with each other in a certain way. Each element is also related to some external elements, and each element of the system has certain functions in the system, while the whole system shows certain functions to the outside. Modern society is extremely complicated, so we must combine the human brain and computers to support each other, so as to form stronger intelligence and create more and newer knowledge [9]. Xiaohua W U believes that bilingual learners will have a positive effect on their cognitive development, while nonbilingual learners will have a negative effect on their cognitive development. Therefore, we believe that in the process of implementing the bilingual education program, when the second language begins to be used as the teaching language, students may be temporarily behind in their studies. When students are proficient in the second language and can meet the teaching requirements, bilingual education will have a positive effect on students' cognitive development [10]. Zhang F believes that teachers should show scientific knowledge by inquiry, and students should learn scientific content by inquiry, use experimental evidence to explain and deepen the content in the textbook, and teach students to use research methods similar to those of biological scientists to process information, that is, to teach students to identify problems and solve them with specific methods [11]. Zou C *X* believes that the digital twin technology learning resources can provide a large number of learning resources for students with its rich and diverse advantages, and the nonlinear organization mode is more suitable for learners' intelligent structure and thinking mode: various information presentation modes are easy to stimulate learning interest; resources have a wide range of radiation, a high degree of sharing, and a fast transmission speed and can be updated in time, which can meet students' demand for resources and is conducive to promoting hierarchical teaching. Students can learn independently according to their different characteristics and situations [12]. Gum believes that the level of students' second language ability depends partly on the level of their first language ability. The hypothesis of dependency reveals the essential difference between proficiency in language and superficial fluency. Proficiency in language means that students have reached the cognitive academic language level, while superficial fluency means that students only have the basic skills of interpersonal communication [13]. *J* believes that the focus of digital education is the construction and sharing of digital resource platforms. A unified learning platform of digital knowledge system should be established, so that different teachers can improve and form their own digital educational resources based on the standardized digital resources provided by the website and better realize the informationization of education [14].

The language goal of bilingual teaching is to gradually make English another suitable medium for teaching and learning in subject teaching. This requires teachers and students to have a certain foundation in listening, speaking, reading, and writing and then gradually develop into the subject field, to enable students to gradually master the special terms and sentences, unique language structures, and expressions of various disciplines, understand the English teaching of the discipline, read the English teaching materials of the discipline, and then communicate orally and in writing on the issues of the discipline in English.

## 3. Introduction of Digital Twinning Technology

### 3.1. The Substantive Significance of Digital Twin Technology

Twinning technology is that any existing or future physical object, system, process, or person is represented by digitalization (digital virtual model), and the state of the physical object is sensed, diagnosed, and predicted in real time by means of the simulation data analysis of the digital model obtained by sensors at any time. The behavior of the physical object is regulated and controlled by optimization and instruction, and the related digital models learn from each other to evolve themselves. At the same time, the manufacturing and decision-making of stakeholders in the life cycle of the physical object are improved, thus improving the production efficiency and reducing downtime. Digital twin technology relies on digital technology to simulate the behavior of physical entities in the real environment and to create a digital mirror image that is completely consistent with the real world [15, 16]. Twin technology can help customers to complete all-digital solutions from product design, production planning, engineering configuration, and manufacturing to service and form a virtual factory based on digital technology.

Research on the application of digital twin technology in the teaching process can broaden and deepen the teaching ideas, improve and optimize students' learning mode, shift from limited empirical learning to digital learning, and avoid the adverse effects of the wrong experience on actual production and processing. The digital twin digital model can easily solve the nonlinear and uncertain factors that the traditional mechanism model cannot solve, improve the production accuracy, and ensure the product quality so that digital twin technology can form an evolving system with machine learning [17–19] and deep learning [20, 21].

### 3.2. Bilingual Teaching Overall Teaching Process Design and Technical Analysis

When Grieves of the University of Michigan in the United States taught a course on product life cycle management in 2003, he introduced the concept of digitalization. The process or method of describing and modeling a physical entity using digital technology that is consistent with its characteristics, behaviors, and performance is referred to as digital twinning technology. It is the actualization of both physical and virtual space. One of the ten strategic technological development trends identified by Gartner is digital twinning. Rosen et al. have investigated a product lifecycle management method, which manages the physical model, virtual model, and engineering data of the product through system integration so that the data related to the product can be fully used in all stages of its lifecycle, and the digital twin technology has made great progress in modeling, simulating, and simulation. As a result, digital twinning is an important application of practical teaching quality evaluation in bilingual teaching, based on the origin and application trend of digital twinning technology. The specific teaching technology analysis is shown in Figure 1.

The concept of bilingual teaching is a higher thinking mode that transcends specific phenomena, the cornerstone of the knowledge content of bilingual teaching, and a kind of knowledge with rationality, abstraction, dominance, and explanatory power. In a certain time and space, the concept of bilingual teaching has typical academic value and can help students solve complex bilingual teaching problems. This paper holds that the effective learning of concepts can be achieved not by simply memorizing, retelling, and applying the names and definitions of concepts but by advanced thinking activities, because concepts are not simple declarative knowledge and skills, and repeated memorizing and intensive exercises cannot help students understand concepts deeply.

### 3.3. Data Support Layer

Compared with traditional teaching, digital twin technology has the advantages of intuition, convenience, quantification, and accuracy. Moreover, digital twin technology can help teachers or students deal with real problems that traditional teaching cannot solve; for example, digital twin technology can “see” bilingual teaching that traditional teaching cannot see. As a means of classroom teaching, digital technology can, on the one hand, establish an intuitive connection between macroscopic phenomena and microscopic essence, effectively reduce the difficulty of content, and thus create a classroom environment that is easy for students to accept. On the other hand, the real-time curve of digital twinning technology can truly reflect the data change process of related parameters in bilingual teaching reaction, promote the formation of students' quantitative view, help students build a knowledge system supported by evidence, and improve their ability to recognize and analyze maps. As an effective combination of information technology and bilingual teaching experiment, bilingual digital twin technology teaching can be used as a teaching method for front-line teachers to choose and use. Twinning technology can record the fleeting experimental data and can analyze and process the data in a multidimensional and comprehensive way, which is beneficial to students' observation and bilingual teaching. Reasonable use of digital twinning technology can achieve the meaningful construction of knowledge and effectively improve the teaching effect of bilingual teaching. It is feasible to use digital twinning technology timely in bilingual teaching concept teaching. The online bilingual teaching system of the digital platform can be divided into the data support layer, modeling, calculation, and simulation layer, function layer, and bilingual experience layer from the basic data acquisition layer to the top application layer. Each layer of the system is closely related to each other, and each layer expands and enriches the functions of the previous layers, as shown in Figure 2.

The digital platform is inseparable from the interaction between reality and virtual teaching space and the perception of things. The data support layer is the key to realizing global stereoscopic perception, and it is the foundation of the whole online bilingual teaching system.

Considering the significance of comprehensive bilingual teaching core literacy, the value of chemical concepts for students' cognitive development, the function of digital experiments in classroom teaching, and the correlation among them, the differentiation of information technology and curriculum integration concept reflects people's different perspectives on the role of information technology. In research and practice, front-line teachers and educational technology researchers agree with the “small integration theory”. Based on the research of experts and scholars and the practice of bilingual teaching, this paper holds that from the perspective of the whole basic education reform, the integration of information technology and curriculum needs to pay special attention to the problems in teaching practice, so the “small integration theory” is more in line with the current development trend and practical requirements. In bilingual teaching, the application of information technology in bilingual teaching in the form of tools is more in line with the reality, as a learning tool for students and a teaching tool for teachers. The integration of information technology in bilingual teaching does not mean that modern teaching media, which is dominated by computer multimedia and network technology, replaces traditional teaching media. Although modern information technology can create a variety of learning environments for students, improve their learning efficiency, become students' cognitive and learning tools, and play an increasingly important role in bilingual teaching, it is still only an element of the bilingual teaching system. Only by integrating it into traditional teaching can it play a greater role.

It can make full use of the school's existing computer equipment, integrate information technology into bilingual classroom teaching, realize the integration, combination, and mutual integration of various bilingual classroom teaching resources, various teaching elements, and teaching links, and enrich, perfect, and expand bilingual classroom teaching under the guidance of the theory of information technology and curriculum integration. It can improve the teaching process in bilingual classrooms, encourage students to learn bilingual classroom content effectively, and encourage the development of innovative talents in bilingual classrooms. Moreover, it can develop students' information literacy, interest in learning bilingual classes, ability to learn bilingual classes independently, and learning habits and methods. It provides a reference for the theoretical and practical research on the integration of bilingual classroom teaching and information technology. It cultivates students' ability to discover, analyze, and solve problems so that they can master the learning style of the information age and have the attitude and ability of lifelong learning; it provides a reference for the theoretical and practical research of the integration of bilingual classroom teaching and information technology. In traditional teaching, textbooks and other media use a linear sequence structure to express knowledge. It takes longer to change because of the difference between people's thinking and knowledge storage modes in learning, the connection between knowledge points in textbooks is not obvious, and the content is limited. The transformation of teaching content presentation and the most effective organization and management of teaching information can be realized by utilizing the hyperlink characteristics of multimedia. They simulate unconditional experiments, difficult-to-observe phenomena, and microstructures in teaching contents with vivid and intuitive images, create and display a variety of realistic learning situations, and integrate abstract learning with real life to improve students' understanding and knowledge of abstract concepts.

With the integration of information technology in bilingual classroom teaching, students are no longer passively accepting knowledge but actively acquiring knowledge. The integration of information technology and curriculum has formed a variety of teaching modes, including lecturing teaching mode, guiding interactive network teaching mode, and research interactive network teaching mode. When students adopt different modes to study or practice, they can not only learn new knowledge according to the teaching contents presented by the computer but also understand and master abstract concepts and some complicated processes through vivid demonstrations so that students can better realize the transition from intuitive feeling to image thinking to abstract thinking through a series of study, observation, and thinking. Students are required to pay more attention to learning methods, thinking methods, and discussion methods and have certain self-learning abilities.

## 4. Analysis of Teaching Effect

This paper makes a statistical analysis on whether there are significant changes in students' information literacy, interest in bilingual teaching, habits and methods of learning bilingual teaching, and ability of autonomous learning bilingual teaching before and after the digital twin technology teaching mode. *Z*-test method is adopted, which is a difference significance test method to determine whether the difference between two averages is significant by comparing the Z-value between two averages with the prescribed theoretical Z-value to see if it is greater than the prescribed theoretical value. This is used to analyze whether the students in the experimental class and the control class have significant changes after a semester of digital twin technology teaching.

### 4.1. Significant Analysis of Overall Capacity Changes

In this section, the back propagation algorithm is used to identify the evaluation system. Its basic idea is the least square method, and the gradient search technique is used to minimize the mean square error between the actual output value and the expected output value of the network. The learning process of the network is the process of correcting the weighting coefficient while the error propagates backward, so it can be used to identify the teaching quality evaluation system, and the input layer is set as shown in formula (2).

(1) $$\begin{array}{c} X=\left\{x\left(1\right),\ldots \ldots x\left(n\right)\right\}, \end{array}$$

where *x* is the evaluation index of the teaching quality evaluation system. The hidden layers of the network are shown in (2) and (3).

(2) $$\begin{array}{c} {\text{net}}_{i}\sum_{j}v_{\text{ij}}X. \end{array}$$

(3) $$\begin{array}{c} O_{i}=a\left({\text{net}}_{i}\right). \end{array}$$

In order to ensure the global stability of the system, the actual output of the identified object (teaching quality evaluation system) is used as a feedback signal, and it is compared with the output of the network identifier. If it does not meet the requirements, the weight coefficient is constantly adjusted to achieve the desired requirements. According to the back propagation calculation formula, the learning rule of the available weight coefficient is shown as

(4) $$\begin{array}{c} a\left(x\right)=\frac{1-e^{-x}}{1+e^{-x}}. \end{array}$$

The output layer of the network is shown as

(5) $$\begin{array}{c} E=\frac{{\left[y-\hat{y}\right]}^{2}}{2}=\frac{e^{2}}{2}. \end{array}$$

The error between the output identification value and the real value of the model is very small. Once the structure of the network and its algorithm are determined, the accuracy of the mathematical model is closely related to the number of input training samples. The three-layer network is used to identify the teaching quality evaluation system, and 10 sample targets are randomly selected. After the training meets the requirements, the identification values shown in Figure 3 can be obtained.

It can be seen from Figure 3 that the original data is very close to the identification value of the network system. The model can accurately determine the teaching effect according to each evaluation index.

This section analyzes the significance of the bilingual teaching model from three aspects, namely, the total average scores of all students before and after the total amount table, the total average scores of all boys before and after the total amount table, and the total average scores of all girls before and after the total amount table. The results are shown in Tables 1 and 2.

From Tables 1 and 2, it can be seen that after the integrated teaching, students' overall ability in information literacy, learning interest, learning habits and methods, and autonomous learning ability have been improved to some extent, both boys' and girls' overall ability has been compared with that before the integrated teaching.

### 4.2. Evaluation of Learning Quality Based on SOLO Classification Theory

After a semester-long teaching experiment, the experimental class and the control class were tested for teaching effect, and the learning quality was evaluated by SOLO classification theory. SOLO classification theory is a theoretical framework of learning quality evaluation put forward by educational psychologist Biggs on the basis of Piaget's structural development theory, which is called observable learning achievement structure. This theory is an evaluation framework composed of five levels; that is, it is composed of five progressive levels: prestructure, single-point structure, multipoint structure, related structure, and abstract extended structure. This theory points out that a person's cognitive structure cannot be detected because of the implicit nature of his overall cognition, but his thinking level when answering specific questions is explicit and can be detected [22]. For the five levels in SOLO theory, the lowest level corresponds to the “prestructure” which refers to students' refusal to answer a question or repetition of a question, the “single-point structure” which refers to students' ability to answer questions with only one isolated clue, the “multipoint structure” which refers to students' ability to answer questions according to multiple unconformized clues, and the “relevance structure” which refers to students' ability to answer questions by linking and integrating multiple clues. Using the independent sample *t*-test to compare the difference in scores between the students in the experimental class and the students in the control class, the suggested results are shown in Figures 4–6.

First of all, by comparing the original data of each student's score on each topic in the two classes, we can know that some students in the two classes can reach the level of SOLO's correlation structure when solving specific problems. However, by comparing the average scores of all students in the two classes, we can know that the average value of the experimental class is between 2 and 3 points, while that of the control class is around 2 points, which shows to some extent that the overall level of the experimental class is near the multipoint structure level and that of the control class is near the single-point structure level. However, neither class has reached the level of the correlation structure. To some extent, it shows that the overall level of the two classes is not very high. Students' ideas are relatively isolated when solving problems, and they have not integrated and summarized the acquired knowledge, thus forming a logical knowledge system.

In addition, from the difference statistics results in Figure 6, it can be seen that the scores of the two classes are compared from the 1st to 3rd questions, and the test results show that the *t*-statistic is 0.412, and the corresponding significance level is 0.684, which shows that there is no significant difference between the students in the experimental class and those in the control class in the learning effect of the 3rd question. From Questions 4 to 7, the independent sample *t*-test of the scores of the two classes shows that the *t*-statistic is 2.337, and the corresponding significance level is 0.214, which has significant statistical significance at a 90% confidence level. It shows that there is a significant difference between the scores of the students in the experimental class and those in the control class on Question 6. From the average, it can be seen that the scores of the students in the experimental class on Question 6 are significantly higher than those in the control class. Comparing the scores of the two classes from Question 8 to Question 10, we can find that there is a significant difference between the scores of the students in the experimental class on Question 8 and those of the students in the control class on Question 8. From the average, it can be seen that the scores of the students in the experimental class on Question 8 are much higher than those of the students in the control class on Question 8. Finally, the scores of the two classes were compared to the total scores. The independent sample *t*-test showed that the *t*-statistic was 3.036, and the corresponding significance level was 0.003, which also had significant statistical significance, indicating that there was a significant difference between the total scores of the students in the experimental class and those in the control class. Further, it can be seen from the average comparison that the total scores of the students in the experimental class were significantly higher than those in the control class.

The results of the second stage test are shown in Figures 7 and 8.

It is found that from the answers of the two classes to Questions 1 to 5, the water average values of the answers of the two classes to the five questions are particularly close. Most students can choose the correct answer to the question, but there is a slight difference in explanation. However, it will not have a big impact on the score, because although the explanation language made by the two classes is slightly different, the SOLO level of the explanation language is the same.

Through the comparative experiment of the bilingual teaching effect of digital twinning technology, it can be found that there are some differences between the average scores of boys and girls in answering questions. The independent sample *t*-test shows that the *t*-statistic is 3.634, and the corresponding significance level is 0.013, which is less than 0.05. It shows that there are significant differences between boys and girls in bilingual teaching in this class of digital twin technology experiment teaching. However, compared with the control class, the results of both boys and girls are higher, so to some extent, it shows that the application of digital twin technology experimental teaching in bilingual teaching will indeed produce certain results.

## 5. Conclusions

The prominent advantage of digitalization is that it can present changing data in time, and this phenomenon requires students to see the essential reasons through intuitive data and requires students to have a better ability to analyze images. The research found that boys' ability to read pictures is better than girls', and digital twin teaching requires students to have a certain ability to understand pictures, so the training effect of digital twin teaching for boys is better than girls'. This also gives a revelation to front-line teachers, who should reasonably and pertinently carry out digital twin teaching according to the cognitive abilities of students of different genders. In addition to different experimental teaching methods, this paper tries its best to keep other factors consistent in classroom teaching. However, there must be other uncontrollable factors that affect the classroom teaching of the two classes, so the research data and results obtained may still be different from the real situation. This paper is an empirical study on the content of two-hour bilingual teaching. This research shows the influence of digital twin teaching and traditional experimental teaching on the learning effect of two-hour bilingual teaching. This is just a practical case. In the future, researchers can carry out comparative studies on other topics, thus more comprehensively explaining the applicability of digital twin teaching [23–25].

## Figures and Tables

**Figure 1:** Analysis of bilingual teaching technology.

**Figure 2:** Online bilingual teaching system based on digital twin platform.

**Figure 3:** Comparison between the original data and the identification value of the network system.

**Figure 4:** Comparison of average scores between experimental class and control class.

**Figure 5:** Comparison of the standard deviation of scores between experimental class and control class.

**Figure 6:** Statistics on the difference in score samples.

**Figure 7:** Comparison of average scores between the experimental class and the control class in the second stage test.

**Figure 8:** Comparison of the standard deviation of scores between the experimental class and the control class in the second stage test.

**Table 1:** Comparison of average score and standard deviation between pretest and posttest.

	Grouping	N	Mean	Mean-difference	Std. deviation
All students	Pretest	201	1.9478	0.1136	0.2192
	Posttest	203	2.0611		0.1384

All boys	Pretest	57	2.0355	0.0238	0.2485
	Posttest	55	2.0582		0.1935

All girls	Pretest	144	1.9138	0.1496	0.1987
	Posttest	148	2.0649		0.1124

**Table 2:** Comparison of significant differences between pretest and posttest.

	*Z*-value	*P* value	Significant degree of difference
All	6.09 > 2.59	0.000 < 0.01	The difference is very significant
Boys	0.662<1.95	0.508>0.06	No obviously different
Girl	6.615 > 2.59	0.000 < 0.01	The difference is very significant

Z-value and *P* value are the parameters of system identification by teaching quality networks.

## Data Availability

The data used to support the findings of this study are available from the corresponding author upon request
